The article "Glutamine Metabolism and Its Role in Immunity, a Comprehensive Review" was retracted in 2021. Reasons: plagiarism; overlap with other authors' work.

# Glutamine Metabolism and Its Role in Immunity, a Comprehensive Review

**DOI:** 10.3390/ani10020326

**Published:** 2020-02-19

**Authors:** Ali Mujtaba Shah, Zhisheng Wang, Jian Ma

**Affiliations:** 1 Key Laboratory of Bovine Low-Carbon Farming and Safe Production, Animal Nutrition Institute, Sichuan Agricultural University, Chengdu 611130, China; alimujtabashah@sbbuvas.edu.pk (A.M.S.); ifraanwar151@gmail.com (J.M.); 2 Department of Livestock Production, Shaheed Benazir Bhutto University of Veterinary and Animal Sciences, Sakrand 67210, Pakistan

**Keywords:** animal, nutrition, metabolism, glutamine, immunity

## Abstract

**Simple Summary:**

Glutamine is a non-essential amino acid, but in disease conditions, it works as essential amino acid and plays a significant role in the animal’s body. Glutamine is a vital amino acid and works to boost immunity in disease conditions and also improves the metabolism in animals.

**Abstract:**

In the body of an animal, glutamine is a plentiful and very useful amino acid. Glutamine consumption in the body of animals in normal or disease conditions is the same or higher than the glucose. Many in vivo as well as in vitro experiments have been conducted to evaluate the importance of glutamine. Glutamine is a valuable nutrient for the proliferation of the lymphocytes. It also plays a crucial role in the production of cytokines, macrophages, phagocytic, and neutrophil to kill the bacteria. Most of the metabolic organs like the liver, gut, and skeletal muscles control the circulation and availability secretion of glutamine. In catabolic and hypercatabolic conditions, glutamine can turn out to be essential and plays a vital role in metabolism; however, availability may be compromised due to the impairment of homeostasis in the inter-tissue metabolism of amino acids. This is why the supplementation of glutamine is commonly used in clinical nutrition and is especially recommended to immune-suppressed persons. Despite this, in catabolic and hyper-catabolic conditions, it is challenging due to the amino acid concentration in plasma/bloodstream and glutamine should be provided via either the oral, enteral or parenteral route. However, the effect of glutamine as an immune-based supplement has been previously recognized as many research studies conducted in vivo and in-vitro evaluated the beneficial effects of glutamine. Hence, the present study delivers a combined review of glutamine metabolism in essential organs of the cell immune system. In this review, we have also reviewed the metabolism and action of glutamine and crucial problems due to glutamine supplementation in catabolic conditions.

## 1. Introduction

Glutamine is an α-amino acid and is the most abundant free amino acid in the body. The first description of glutamine importance was by Ehrensvard et al. [1], who described the importance of glutamine in cell survival and proliferation. In the body of an animal (cells and tissue), the amino acid is a building block and the second most important and abundant compound after water. The animal body itself can produce most of the amino acids, or they can be obtained from the diet, and the availability of these amino acids is vital for the production and survival of the body of the animal (cells) and proliferation. Specific animals have developed different pathways (biochemical and metabolic) to resist the infection-causing pathogen through enhancing the catabolism of amino acids to help immune reaction, therefore limiting the availability of nutrients that contain nitrogen to attack the microorganism [2]. Thus, for a host, this evolutionary mechanism is beneficial for controlling the inflammatory response to infection.

The article "Glutamine Metabolism and Its Role in Immunity, a Comprehensive Review" was retracted in 2021. Reasons: plagiarism; overlap with other authors' work.

Among the 20 amino acids, glutamine is important and plays a key role in the amino acid metabolism and also performs a vital role in immunity against pathogens. In an animal’s body, glutamine is a useful amino acid that is present in rich form and is important for intermediary metabolism, and the exchange of nitrogen through transportation of ammonia between tissues and homeostasis. Glutamine can be used in all the cells as a substance for the production of nicotinamide, adenine phosphate, nucleotides, purines, pyrimidine, antioxidants, and numerous additional biosynthetic pathways concerned in the integrity of cells and their normal function [3]. 

For the normal function of the body cells, most of them require nutrients; however, in the immune system, the cells perform their role in the nutrient-restricted microenvironment [2]. Although in the body, glucose is a most important metabolite and primary fuel for cells, immune cells (lymphocytes, neutrophils, and macrophages) utilize higher or equal rates of glutamine compared to glucose in catabolic conditions like recovery from surgery burns, sepsis, undernutrition and physical exercise [4,5]. In the 1980s, the laboratory of Eric NewShelome, the University of Oxford and many other institutes all over the world extensively acknowledged this theory (1935–2011). Based on their hypotheses, the idea of “immune-metabolism” [3,6,7,8,9], the current motive immune system used the glutamine amino acid as a fuel for their proper function; in addition, the low level of blood may damage the role of immune cells, subsequently developing poor clinical consequences and an up-surged in the death rate [10]. Presently, glutamine is generally used in clinical nutrition, supplementation in pre- and post-operative patients and also used by athletes to restore their immune functions.

The article "Glutamine Metabolism and Its Role in Immunity, a Comprehensive Review" was retracted in 2021. Reasons: plagiarism; overlap with other authors' work.

## 2. Glutamine Metabolism

The molecular weight of glutamine amino acid is 146.14 g/mol, with five carbons and the compositions of its elements are 41.09% carbon, 6.09% hydrogen, 32.84% oxygen, and 19.17% nitrogen. According to its pH, glutamine (amino acid) is classified as neutral while glutamine is a non-essential amino acid based on its nutritional properties. Commonly, two amino groups are present in glutamine, the α-amino group and the amide group (simply hydrolyzed side chain), and such features of glutamine facilitate its vital role as an ammonia carrier and nitrogen transporter; it has also been noticed that glutamine has properties enabling it to combine with protein [9].

A healthy human being (average 70 kg body weight) has about 70% to 80% glutamine disseminated in the whole body [11]. According to the pharmacokinetics and isotopic methods, it has been assessed that per day, endogenous glutamine synthesis is about 40–80 g in a normal person [12,13]. On the other hand, in the fasting stage, the glutamine concentration is about 500–800 µM/L, in blood plasma samples and this indicates that in the blood, nearly 20% pool of the amino acid is present [9]. In the tissue, skeletal muscles and the liver, the concentration of glutamine is much higher than the plasma; it accounts for 40–60% of the total amino acid pool [14,15]. Glutamine is considered as the most plentiful amino acid of the animal body because in plasma and body tissue, the glutamine level is 10 to 100 times higher than any other amino acid. In the body of animals, the glutamine level depends on the production and utilization of body/uptake by different organs and tissues. Most of the glutamine synthesis occurs in the brain, liver, lungs, adipose tissues and skeletal muscles. In contrast, the organs which have a more significant glutamine activity, degrading capacity and consumption rate are leukocytes, intestinal mucosa, and renal tubules cells. Nevertheless, in the reduced carbohydrate concentration in muscles [16]/amino acid uptake [17], disease/stress condition, the muscle tissues produce less glutamine and the liver consumes more glutamine [16]. Numerous additional factors, mostly Thyroid [18,19] growth hormones [19] glucocorticoid [20] and insulin, can reduce the activity of metabolism-regulating enzymes of glutamine.

In the metabolism of glutamine, various enzymes are involved, such as phosphate-dependent glutaminase (GLS) and glutamine synthetase (GS). GLS is accountable for the hydrolysis of glutamine, which transforms it into glutamate-ammonia ions NH_4_ again, while the GS is activates the reaction which produces glutamine ammonia ions NH_4_ [21,22] (Figure 1). In the intercellular space, the GS is mainly present in the cytosol; however, GLS inactive farms are mostly present in the mitochondria. These sites are compatible with the functions of enzymes; GLS in the tricarboxylic acid cycle (TCA) catalase glutamine conversion to glutamate entry at 2-oxoglutarate as a source of energy or foundation of metabolic intermediates [6].

The article "Glutamine Metabolism and Its Role in Immunity, a Comprehensive Review" was retracted in 2021. Reasons: plagiarism; overlap with other authors' work.

The availability of glutamate is necessary for the synthesis of glutamine through GS. Glutamate is synthesized by the action of glutamate dehydrogenase from the two oxoglutarate NH_4_ or another amino acid, leucine (branched-chain amino acid) catabolism [17,23]. Research evaluating leucine in rodents has found that transmitted with ketoglutarate to synthesize glutamate, it can integrate free ammonia and the activity of the GS can synthesize glutamine [5,23] (Figure 2).

In the blood and tissue, the concentration of glutamine depends on the functions of GS and GLS. In a catabolic condition such as Sepsis [3,24], surgeries [8] trauma [10] infection [25,26] as well as during prolonged exercise [27], the endogenous synthesis of glutamine does not fulfill the requirements of the human body. Glutamine assumes the role of essential amino acid sometimes in such deficit situations through increasing expressions of GLS and reduces the function of GS [14]. However, it is worth highlighting that the concentration of glutamine in plasma is decreased from its normal range of 500–800 µmol/L to 300–400 µmol/L because as cells depend on glutamine, so the lower concentration affects the immunity cells, in terms of function and proliferation [5]. Conversely, higher catabolism of tissue leads to a decrease in the stock of glutamine in human tissue, mostly in the liver and muscle. Low levels of glutamine in the tissue of a human influences the entire body; meanwhile glutamine offers atoms of nitrogen for the formation of amino sugars, purines and pyrimidines [28]. If glutamine deprivation in these tissues continues, the mechanism and considerable number of metabolic pathways which depend on the availability of glutamine are affected, and as a result, suppression of immunity occurs. In addition, the currently, research has reported that infections that are caused by bacteria such as Escherichia coli could change its harness and glutamine metabolism to suppress the influence of copper toxicity and acid stress [29]. Therefore, pathogens can adapt and persist through changing the central metabolic pathways, which is vital for host protection against the bacterial attack. 

The article "Glutamine Metabolism and Its Role in Immunity, a Comprehensive Review" was retracted in 2021. Reasons: plagiarism; overlap with other authors' work.

## 3. Immune Cells Function and Glutamine

In 1873, glutamine was first considered as the essential biological molecule when some indirect testimonies described it as a protein structural constituent; then, in 1833, copious amounts of free glutamine was found in some plants. After the study of Hans Adolf Krebs in 1930, further research studies were conducted. In 1930, Sir Kreb found, for the first time in the history of science, that glutamine can be hydrolyzed and produced by mammalian tissue [21,30]. Eagle et al., in 1950, found that in the cell incubation period, isolated fibroblast utilizes a higher amount of glutamine than any other amino acid. Additional research in this period was hindered due to the classification of glutamine as a non-essential amino acid and the fact that it was very hard to calculate the concentration of glutamine in tissues and plasma.

Glucose is a vital metabolite which is essential fuel for body cells; during the 1980s, Eric Newsholme concluded that glutamine is an important modulator for the function of the leukocytes, for example, macrophages [31] and lymphocytes [7]. Newsholme P. et al. [31] reported that macrophages actively use glutamine. Moreover, Pithon Curi et al., in 1997 [32,33], reported that neutrophils use glutamine. The research of Eric (Lymphocytes) and Philip Newsholme (macrophages) on metabolism encouraged numerous other publications, which increased from two to three papers per year from 1960 to 1970 to about more than 50 research publications in the past 20 years.

During high catabolism and disease conditions, the glutamine utilization by the cells is higher or equal to the glucose utilization [34,35] so in such circumstances, the use of glutamine is increased by the tissues and the liver, which leads to a shortage of glutamine in the body of animals. Furthermore, glutamine is produced in the skeletal muscle of the animal’s body, which decreases their ability to manage the level of glutamine in plasma (Figure 2). 

Glutamine in immune cells is converted into glutamate, alanine, and aspartate through partial oxidation of the carbon dioxide (glutaminolysis), while glucose is converted into lactate through glycolysis [6] (Figure 2); this alteration is a vital part in the function of the immune system. Glutamine degradation and aspirate ammonia formation lead to the production of purine and pyrimidine in deoxyribonucleic acid and ribosomal nucleic acid. Glutamine present in the body acts as a vital part of the immune cells’ gene expressions [6], such as the proliferation of immune cells controlled by glutamine through the activation of the extracellular signal-regulated kinase (ERK) and c-Jun N-terminal kinases (JNK) kinases proteins. These proteins activate the transcription factors JNK and activator protein 1 (AP-1) and cause transcriptions of the genes related to cell proliferation. In connection, the suitable level of glutamine enables the surface markers of the primary lymphocyte cells, for example, CD25, CD45RO and CD71 and also the synthesis of the cytokines (IFN-γ, TNF-α, and IL-6) [28,36,37,38]. Hence, Glutamine plays a vital role in cell proliferation and leukocyte uses glutamine as an energy substrate and also contributes to the process of tissue repair [39].

The article "Glutamine Metabolism and Its Role in Immunity, a Comprehensive Review" was retracted in 2021. Reasons: plagiarism; overlap with other authors' work.

## 4. Neutrophils

Glucose is the chief subtract for the existence and generation of reactive oxygen species (ROS) and endocytosis for neutrophils. However, as an energy metabolite, glucose is not the only source of energy for these cells. Interestingly, neutrophils utilize more glutamine than other leukocytes such as lymphocytes and macrophages [40]. In neutrophils, most of the glutamine is converted into aspartate, glutamate, and lactate through the Krebs cycle. For the proper function of leukocytes and the generation of vital compounds, including Glutathione (GSH) and its metabolism, glutamine, glutamate, and Carbon dioxide play an essential role in favorable conditions. Neutrophils use structural proteins which have chromatin (uncondensed) and antimicrobial factors known as neutrophilic extracellular traps (NETs). NETs need the formation of ROS, enzyme production (Myeloperoxidase and elastase) and other compounds capable of killing extracellular bacteria and overriding the virulence factors [41]. The mechanism requires ROS to turn on the initiation of the nicotinamide adenine dinucleotide phosphate oxidase (NADPH) oxidase 2 complex. Regarding glutamine, for the synthesis of malate, the malic enzyme is used for the production of a higher quantity of NADPH; meanwhile, NADPH is essential for the synthesis of superoxide anion (O_2_^−^), which represents action against the microbes. Likewise, glutamine is also used by the macrophages for arginine and consequently, the synthesis of nitric oxide via the activity of enzyme-inducible NO synthase (iNOS) through utilizing NADPH as a source of energy. In the neutrophil, glutamine enhances the production of superoxide by the activity of NADPH oxidase.

Furthermore, an inhibitor phosphate dependent on glutamines, known as 6-Diazo-5-oxo-l-norleucine (DON), which inhibits the metabolism of the glutamine, causes a decrease in the synthesis of superoxide through stimulation of the neutrophils with phorbol myristate acetate (PMA). PMA increases p47, p22, and gp91 mRNA expressions and is a crucial constituent of the NADPH oxidase complex. Glutamine increases the expressions of these three proteins in the presence or absence of the PMA. In the neutrophil, glutamine increases the production of the superoxide through the synthesis of adenosine triphosphate (ATP) and regulates the expression of a component of the NADPH oxidase complex [42]. The action of glutamine is important to avoid alteration in the activity of NADPH oxidase and the generation of the superoxidase prompted by adrenaline in neutrophils [43]. 

The article "Glutamine Metabolism and Its Role in Immunity, a Comprehensive Review" was retracted in 2021. Reasons: plagiarism; overlap with other authors' work.

## 5. Macrophages

During the macrophages’ activation process, the glucose and glutamine metabolism is greatly affected [44,45]. The effects of activation stimulus Bacillus Calmette Guerin (BCG) and an inflammatory stimulus thioglycollate on the metabolism of glutamine and glucose in macrophages have already been studied by [46]. Either BCG or thioglycollate increases the action of citrate synthase and hexokinase and the oxidation of the glucose while BCG noticeably enhances the glutamine metabolism. The metabolism of glutamine and glucose is involved in polarizing signals that increase the transcriptional program needed in the capacity of macrophages to perform a particular function. In the metabolic pathway and related signalling activation, protein kinase B, the mammalian target of rapamycin (mTOR) complex and AMP-activated protein kinase play a crucial role [47,48]. Extracellularly available glutamine may have a part in the regulation of mTORC1 through particular nutrient-induced starvation [17]. The production and secretion of pro-inflammatory cytokines (IL-6, IL-1, and TNF) through macrophages are also controlled by the obtainability of glutamine. Numerous types of macrophages (M1 and M2) have been recognized [49,50]. M1 and M2 macrophages are formed due to the reprogramming of signalling pathways; this reprogramming change in the signalling pathways in macrophages involve alteration in the metabolism of glucose and glutamine [51]. No study has recognized that the fatty acids required for the polarization induced human IL-4 macrophage [52]. This issue, however, remains controversial. Macrophages change their function and metabolism for the polarization of anti-inflammatory cells, due to stimuli and ecological circumstances [53]. Glucose-dependent oxidative phosphorylation of aerobic glycolysis (Warburg effect) occurred when macrophages were treated with Lipopolysaccharide (LPS). IL-1β expression and hypoxia-inducible factor 1-alpha (Hif-1α) activity is regulated by pyruvate kinase M2, which is a significant molecule to encourage the Warburg effect in macrophages (activation of LPS) [54]. Owing to this mechanism, M1 macrophages display a rapid enhancement of the formation of ATP, which is needed for the defense mechanism of the host [51,55,56]. M2 macrophages in the TCA cycle have no metabolic escape flux while LPS-treated macrophages M1 have two substrate flux deviations, one at the formation of the post succinate and the other during the reaction of the isocitrate dehydrogenase step. As a result, there is a formation of succinate, citrate, ketoglutarate, and itaconate (TCA cycle intermediates) that controls the activation of the LPS macrophage [56]. For the alternative activation of macrophage (IL-4), glutamine is required [57,58]. Through glutaminolysis, the alpha-ketoglutarate is generated; thus, it endorses the differentiation of macrophages M2 [59,60] peroxisome proliferator-activated receptor (PPAR alpha) which has been reported to be needed for glutamine oxidation, gene expression (IL-4) and to stimulate the respiration of a macrophage. Therefore, the metabolism of glutamine plays an essential role as a modulator and synergetic supporter for the activation of a macrophage. 

The article "Glutamine Metabolism and Its Role in Immunity, a Comprehensive Review" was retracted in 2021. Reasons: plagiarism; overlap with other authors' work.

## 6. Lymphocyte

The activation of the lymphocyte function depends on a specific metabolic pathway. In CD4 + T cells, signalling pathways and transcriptional programs are affected by multiple extracellular signals, such as different events consisting of a change in energy metabolism, the production of cytokines, and the proliferation of cells. Related bioenergetic procedures are contingent on activated protein kinase (AMPK) activation, showing a link between the signalling pathway and metabolism in the differentiation of immune cells. In the thymocytes of a rat, glycolytic pathway (anaerobic) usage has highly increased the stimulation of antigen with concanavalin afterward. Eric Newsholme’s group were the first to report that glutamine was utilized by the lymphocytes [61]. It has been noticed that glutamine plays a crucial role in the different functions of these cells. The metabolism of glutamine and glucose in cell pyruvate is a common product. Curi et al. [62] reported that Mesenteric lymphocytes have greater pyruvate oxidation by pyruvate carboxylase when stimulated with concanavalin, showing that glutamine and glucose are implicated in the function as well as in the proliferation of lymphocytes. The mitochondria control the activation of leucocyte. Different metabolites of the Kreb cycle which are produced during the metabolism of glutamine and glucose, such as citrate, fumarate, and succinate, take part in inflammation control and immunity in both adaptive and innate immunity [39].

Copious amounts of glucose molecules are transferred through glucose transporter 1, whereas this has not been noticed in non-activated lymphocytes [63]. In the activation of lymphocyte, glucose transporter 1 is a vital metabolic marker which rapidly transfers to the surface of the cell after stimulation [64]. Wieman et al. [64] further reported that CD4+ T cells produce a more significant amount of TNF, INF, IL-2, IL-4 and lower basal proliferation rate due to glucose deficiency. Intracellular signalling activation by Akt beyond GLUT1 concentrations of protein leads to more upsurges in the uptake of glucose and T cells activation. In immunity and metabolism, mTOR and AMPK act as an essential role. Lymphoid cell activation leads to the upsurge of GLUT1 uptake of glucose by acting on the mTOR protein [65]. The current metabolic process takes part in the differentiation of CD4 as well as in T cell subunits, as mTOR-deprived mice show reduced differentiation for effector T lymphocytes [66,67]. Moreover, the AMPK cycle suppresses mTOR via and has a blocking effect on the signalling of this protein, leading to the initiation of oxidative metabolic pathways rather than the glycolytic pathway within mitochondria [68,69]. The proliferation process of T and B lymphocytes along with the generation of protein, synthesis of IL-2, and synthesis of antibody rates require glutamine. Numerous research studies have shown that the metabolism of glutamine plays an important role in lymphocyte activation.

The article "Glutamine Metabolism and Its Role in Immunity, a Comprehensive Review" was retracted in 2021. Reasons: plagiarism; overlap with other authors' work.

ATP is required for the expenditure of higher energy, while the forerunner is needed for the synthesis of complex molecules, for example, nucleotides and lipids for DNA and RNA synthesis in the cell proliferation process. To accomplish the quick activity of proliferation below a certain amount, lymphocytes change from oxidative phosphorylation to glycolysis (aerobic) and glutaminolysis, and thus, noticeably upsurge glutamine and glucose consumption. In the lymphocyte, the transition of the metabolism is vital for T cells activation; meanwhile, the metabolism of glucose delivers intermediates for the biosynthesis pathways, which is necessary for differentiation and growth of the T cells [70]. Glycolysis plays a vital part in the function of effector T cells related to inflammatory cytokines production, mostly IL-2 and INF-a [71]. Thus, a higher glycolytic activity is related to Th0 and Th1 cells differentiation [68]. The glycolytic pathway inhibition will block this process while increasing the differentiation of Treg cells. Proliferating cells increase glycolysis, which ultimately increases the uptake of glucose and also increases the activity of glycolytic enzyme and expression while the utilization of glucose in the pathway (oxidative phosphorylation) is reduced. Thus, metabolic switch requires greater energy; the formation of macromolecules and suppression of metabolic futures of rest lymphocyte require the production of metabolic intermediates. Insufficient delivery of nutrients or particular inhibition of the metabolic pathway prevents the proliferation and activation of T cells and subsequently, the incapability to utilize glucose prevents differentiation of T cells in vivo and in vitro [70,72]. The function and metabolism of T lymphocyte are closely related to mitochondria dynamics. The active T cells effectors have a punctuated region and also enhanced anabolic activity. Moreover, these memory T lymphocytes possess fused mitochondria with energetic oxidative phosphorylation activities [73]. In the activation of T cells and the maturation of dendritic cells, the hypoxia-inducible factor 1-alpha (HIF1-α) plays a critical role. This factor controls the metabolism reprogramming of leukocyte by altering its gene expression and thus, functions of immune cells [74].

The article "Glutamine Metabolism and Its Role in Immunity, a Comprehensive Review" was retracted in 2021. Reasons: plagiarism; overlap with other authors' work.

Active T cells effectors have a punctate mitochondrial region and enhanced anabolic activity. Moreover, the memory T lymphocytes fuse mitochondria with strong oxidative phosphorylation activities. Glutaminolysis and glycolysis are related to ensuring the proper functioning of the lymphocyte. Hexosamine biosynthesis requires glutamine and glucose for uridine diphosphate N-acetylglucosamine de novo production. The nucleotide prevents signalling and receptor endocytosis by encouraging the branching of Asn (N)-linked glycans (N acetylglucosamine). Reference [75] described that the more significant aerobic activities of glutaminolysis and glycolysis are a helpful way to reduce the synthesis of UDP-GlcNAc and branching of N-glycan in blasts of T cells in the mouse, because of the reduced accessibility of these metabolites for the synthesis of hexosamine.As a consequence, growth and pro-inflammatory TH17 features prevail over anti-inflammatory-induced T regulatory (iTreg) differentiation. The last function is endorsed by IL-2 receptor alpha loss by endocytosis. The researchers formerly assumed that a primary purpose of attendant greater glutaminolysis and glycolysis (aerobic) function is to control precursors in the biosynthesis of N-glycan. The current metabolic prospect of T lymphocyte has noticeable insinuation in cancer and autoimmunity. It has also been noticed that for the formation of polyamines, spermine, spermidine, and putrescine glutamine play a critical role as precursors. Higher concentrations of polyamines are found in autoreactive B and T cells in autoimmune disease and tumor cells. For normal immune cell function and also in related properties of anti-tumor immune cells and autoimmunity, polyamines play a vital role [75].

The article "Glutamine Metabolism and Its Role in Immunity, a Comprehensive Review" was retracted in 2021. Reasons: plagiarism; overlap with other authors' work.

## 7. Clinical Application of Glutamine Supplementation

Glutamine amino acid has metabolic rules; glutamine seems to have major potential in normal animal production systems as well as in disease conditions. In practice, however, responses to the supplementation of glutamine have been inconsistent. Therefore, in ruminants, during lactation and growth studies, both positive and null effects on production responses have been noticed [76]. Likewise, therapeutic responses of glutamine supplementation during several digestive tract disorders have been inconsistent in both ruminants and pigs. This is despite the proven connection that nucleic acid biosynthesis is essential to support cell proliferation. In sheep, at least, glutamine may exert a protective effect against hepatic amino acid (AA) oxidation, mainly for methionine. This may suggest an anabolic potential because methionine is the main limiting amino acid in a number of animal feedstuffs. Glutamine is also vital in control of metabolic acidosis, but, in contrast to rodents, the key site of production seems to be extra-hepatic [76].

The supplementation of glutamine is mostly used in patients who have clinical findings such as burns, trauma and following injuries. In severe metabolic stress, the production of glutamine is increased and released to fulfill the requirement of the metabolic demand for faster dividing cells, for example, in the immune system and in the gastrointestinal tract [77]. Glutamine amino acid reduction may contribute to weight loss, infection and muscle wasting in trauma and seriously ill patients [78]. These findings have been proposed as an argument for glutamine supplementation. Various randomized research studies reported that supplementation of glutamine has a positive effect on various organs and systems in the body [79,80]. Furthermore, some studies confirmed that the administration of glutamine through the parenteral route has no adverse effect on the health and does not cause any change in the central nervous system, including in blood chemistry [81]. The researchers also described a greater concentration of glutamine within five days after treatment with glutamine [82]. Likewise, no side effect was observed when elective abdominal surgery was performed with the administration of 0.285 g/kg body weight glutamine increased total parenteral nutrition [82]. Indeed, glutamine supplementation improves the nitrogen balance and intramuscular sparing glutamine pool [82]. In addition, some studies reported that enteral feeding is a method of choice to increase the level of glutamine in systemic circulation. In fact, research in healthy individuals proposes that 40–50% of radiolabeled glutamine enters the circulating pool, whereas the residual 50–60% is used by the splanchnic bed [81].

The article "Glutamine Metabolism and Its Role in Immunity, a Comprehensive Review" was retracted in 2021. Reasons: plagiarism; overlap with other authors' work.

## 8. Conclusions and Future Viewpoints

Glutamine is required for the proper function, proliferation, and survival of immunity cells, and eventually, these cells protect the animal’s body against various pathogens. The demand for glutamine is dramatically increasing in catabolic and hyper-catabolic conditions; sometimes, these conditions cause deprivation of glutamine in the body and impair the immunity function. However, the level of glutamine did not decrease in all catabolic states or severely ill patients, and consequently, no everyone will get the beneficial effects of glutamine supplementation. It is necessary for glycemia to maintain the constant levels of glutamine in plasma glutamine and inter-tissue metabolic flux, especially for the high catabolism activity of organs, such as liver, skeletal muscles, and gut. Not astonishingly, the conditions of a lower level of glutamine and its severity are different between animal and human research, and in themselves, do not deliver a rational argument for the supply of exogenous glutamine. In certain catabolic conditions and when there is glutamine shortage from the diet, amino acid supplementation is required. Incidentally, the effectiveness of glutamine supplementation in immunity have been comprehensive researched and novel queries and viewpoints are being expressed. For illustration, future work should evaluate the nutritional intervention frequency, ideal amounts related to stress or disease conditions, and associated administration with dipeptide mixtures or other amino acids. Furthermore, the developing era of metabolomics has the possibility to increase our sympathy toward the multifaceted regulation of the metabolism of glutamine, recognizing new metabolites such as Itaconate in macrophages which are crucial for cell function and are therefore more effective than the idea of “the fuel for the immune system.”

## Figures and Tables

**Figure 1:** Synthesis and hydrolysis of Glutamine. Glutamine is mostly synthesized and hydrolyzed through the enzymes glutamine synthetase (GS) and glutaminase (GLS), respectively. GS catalyzes glutamine biosynthesis through ammonia and the glutamate source. In response, one adenosine triphosphate (ATP) is utilized. Many amino acids (exogenously or endogenously) provide the glutamate through catabolism. Moreover, GLS is responsible for the hydrolysis of the glutamine and the formation of glutamate and ammonia ion (NH_4_). Nearly all body cells express GLS and GS and their primary expression and function is carried out if the tissue is more likely to synthesize or utilize the glutamine in normal or disease conditions.

The article "Glutamine Metabolism and Its Role in Immunity, a Comprehensive Review" was retracted in 2021. Reasons: plagiarism; overlap with other authors' work.

**Figure 2:** Glutamine production and utilization inside the tissue in health and disease conditions. The blue arrows designate tissue that shows the activity of GS and thus, the synthesis of glutamine; The white arrows designate tissue that shows the activity of GS and thus, the utilization of glutamine. In healthy or in fed conditions, glutamine stocks are equal in plasma and tissues and are sustained mostly by the liver and skeletal muscles. There are two major sites for the storage of glutamine in the body. Alternatively, immune cells enormously depend on glucose and glutamine in condition (**A**), and more in condition (**B**). While the GIT is a principal place for the utilization of the glutamine in condition (**B**), glutamine utilization from both the basolateral and luminal membranes is increased when compared to condition (**A**). Furthermore, the liver changes its role from chief glutamine producer to chief glutamine consumer to sustain gluconeogenesis and the entire body depends on the skeletal muscle’s ability to sustain the glutamine concentrations. The current reaction is typically accompanied by a dramatic upsurge proteolysis of muscle, cachexia, and atrophy. The adipose tissue and lungs exhibit enzymes GS and GLS, and hence, can synthesize and utilize glutamine in conditions (**A**,**B**). The kidneys and brain do not exhibit GS, only GLS, and hence, are mostly reliant on the availability of plasma glutamine in conditions (**A**,**B**).
